# Systematic Evaluation of the Effect of Rehabilitation of Lower Limb Function in Children with Cerebral Palsy Based on Virtual Reality Technology

**DOI:** 10.1155/2021/6625604

**Published:** 2021-03-08

**Authors:** Chao Gao, Yongli Wu, Junting Liu, Runhan Zhang, Manting Zhao

**Affiliations:** Cangzhou Central Hospital, Cangzhou 061000, Hebei, China

## Abstract

As times go by, people's standard of living is constantly improving, but the medical pressure exerted by children with cerebral palsy is also increasing and the recovery of lower limb function in children with cerebral palsy after treatment has also gets people's attention. Of course, the relevant medical equipment is constantly improving, especially the appearance of virtual reality technology, which has played an extremely important role in restoring the lower extremities of children with cerebral palsy. In order to study the role that virtual reality technology can play in children with cerebral palsy, this article collects relevant information, builds a case template, and uses comprehensive quantification by investigating patients, examining relevant documents, and interviewing professionals. With qualitative analysis, a damage assessment matrix is created. Experimental results prove that the use of virtual reality technology can improve the treatment efficiency of children with cerebral palsy by more than 30%. In terms of the rehabilitation effect of children's lower limb function, virtual reality technology is more targeted for the treatment of children with far-reaching effects. It is much higher than traditional treatment methods, and the mobility of the children's lower limbs is restored by more than 80%. This shows that virtual reality technology can play an important role in the rehabilitation of the lower limbs of children with cerebral palsy.

## 1. Introduction

With the continuous improvement of my country's medical service system, the rehabilitation of lower limb function in children with cerebral palsy has received more and more attention [1]. Sport rehabilitation is an important sector of medical rehabilitation and the most widely accepted work in the social security system. In the process of continuous improvement of restoration services, the restoration industry based on virtual reality technology is moving towards production, industrialization, and individualisation. Virtual reality technology provides a great help for the rehabilitation of patients [2]. Virtual reality technology can be traced back to the late 1980s. It is a kind of comprehensive manufacturing technology that has subverted the traditional manufacturing process and has a brand-new thinking mode that has gradually emerged since then. It is based on software technology, machining technology, and special processing technology, micromolecular science, and electrical and electronic technology as its foundation. Virtual reality technology is a revolution to traditional manufacturing technology and provides a new platform for its development [3]. Compared with the traditional manufacturing technology in the past, virtual reality technology can not only realize “from scratch” and save a lot of time and labor [4] but also carry out “personalized manufacturing” to make the product unique. At present, the medical industry is generally concerned about virtual reality technology. It has achieved good results in the experimental demonstration of new product development, rapid mold making, and direct production of small batches of special complex parts, bioengineering applications, and the development of new materials [5]. This technology can quickly deliver abstract and complex ideas in design innovation. It can be constructed in a way, to save materials and reduce energy consumption. It can use graphical or animated drawings to express the rapid process of manufacturing individual products and to show people in the future its tendency, the search for differentiated and individualised products. It can be used in the form of graphical cases to show the functions and functions of integrated design and optimised design and construction [6]. There are also many domestic and foreign research studies on the role of virtual reality technology in the rehabilitation of lower limb function of children with cerebral palsy.

In order to evaluate the effect of virtual reality technology on the rehabilitation of upper and lower limbs of stroke patients, Yang Yujie used computers to search major databases, such as HowNet and Wanfang, to research the related literature and to systematically analyze literature data using computer software. He concluded that virtual reality technology has a significant effect on the rehabilitation of upper limbs of stroke patients, but it is not obvious for the rehabilitation of patients' lower limbs [7]. Cheng Xiuyan analyzed the application of virtual reality technology in medical treatment, especially in stroke patients, and the use of virtual reality technology can allow patients to better maintain their recovery function. It has designed experiments on the clinical data of the hospital in recent years and performed virtual reality technology treatments on patients for several weeks. Comparing the parameters of these skills with patients undergoing traditional treatment methods, it is concluded that virtual reality technology can effectively improve the patient's lower extremity balance and is conducive to patient rehabilitation [8]. Xu Lei, in order to evaluate the impact of virtual reality technology on patients with cerebral palsy, created a three-dimensional gait analysis system, divided patients into groups, and performed different treatments on patients [9]. After a certain treatment time, the patient's stride length, stride frequency, and other important indicators for cerebral palsy patients are tested. Experimental results prove that virtual reality technology has a good effect on the patient's walking ability [10]. These studies have improved the relevant reference role for this article. However, due to insufficient samples of these studies, too much emphasis on theories, and unreasonable practical schemes, the research has too many variables and the conclusions are unconvincing.

This article analyzes the advantages and disadvantages of the previous research and then proposes a model of the rehabilitation efficacy of lower limb function in children with cerebral palsy based on virtual reality technology. This article mainly describes the basic characteristics of the impairment of the ability of the lower limbs in children with cerebral palsy, and the composition is described in four aspects: grid, individual definition, status, and action definition and interaction between individuals. The system objectively assessed the clinical relevance of restoring the function of the lower limbs in children with cerebral palsy, explained the damage of children with cerebral palsy in patients, and verified the role of virtual reality technology in the treatment of children with cerebral palsy.

## 2. Rehabilitation Treatment Methods of Lower Limb Function in Children with Cerebral Palsy

### 2.1. Virtual Reality Technology

The continuous development of virtual reality technology has deepened the connotation of virtual practice. In essence, the practice of virtual reality technology is still transforming things in objective reality into digital image symbols through photoelectric and other means, and then expressing them in virtual space come out [11]. However, difference from the usual virtual practice is that the practice in virtual reality makes the practice subject completely immersed in a virtual environment that can get real feelings, and through sophisticated sensing technology, people can obtain vision, hearing, touch, and smell that are the same as reality. And the comprehensive feeling of kinesthesia and then the motion tracker of various parts of the human body will feedback the subject's feedback into the virtual space and cyclically interact [12].

Virtual reality technology has brought about changes in human working life, entertainment, and practical methods. At the same time, it also caused social problems such as excessive leniency, health effects, violence, and value orientation, and the development of the field of philosophy was born. The traditional philosophy of technology tends to study the various social effects of technology, but at the same time, the development of technology will also have an impact on the philosophy system. Affected by virtual reality technology, branches of philosophical fields such as artificial intelligence philosophy, virtual reality philosophy, and artificial life philosophy continue to appear. The philosophical issues generated by virtual reality technology involve many fields such as practical theory, media theory, epistemology, ethics, and sociology. Its unique technical characteristics and practical methods have produced different depths of utility in multiple disciplines [13].

The characteristics of virtual reality technology make philosophers pay more attention to some traditional philosophical theories, such as the study of ontology and thinking about the nature of the world. Some brand-new philosophical ideas have emerged at the historic moment. In view of the technical characteristics of virtual reality that can construct a brand-new virtual environment, some scholars have put forward the idea that “computing” is the essence of the world. For example, the American philosopher Steinhart proposed digital metaphysics. Zhai Zhenming, a philosophy professor at Sun Yat-sen University in my country, proposed a new ethics “world-making ethics” and so on. Facing the continuous innovation of technology, philosophical thinking cannot stop but should lead and correct the new technology [14].

Since the advent of the Internet, virtual practice has attracted much attention. Through virtual practice, mankind has broken through material production practice, social practice, and scientific practice, expanded the scope of practice, increased the objects of knowledge, and improved the practical ability. The development of virtual reality technology has added new vitality to virtual practice. If virtual practice is a practice that creates possibilities, then virtual reality practice is a practice that transforms any possibility into reality. In the virtual environment, any condition becomes controllable, and human beings are no longer restricted by physiological, natural, and social factors and get rid of the shackles of material conditions [15]. The digital symbols with bits as the unit abstract the original concrete things. In reality, the function of things is separated from the material carrier of the thing, and its function can be used alone anytime and anywhere without being restricted by the material carrier. This is no exception for people. Virtual reality pulls human senses and consciousness out of the body, realizing truly beyond the limitations of time and space. For the application of virtual reality technology in medical treatment, we generally adopt the following formula:

(1) $$\begin{array}{c} x\left(k+1\right)=Ix\left(k\right)+Jv\left(k\right),\;k=1,2,\ldots . \end{array}$$

The quadratic performance indicators are as follows:

(2) $$\begin{array}{c} K=\sum_{k=1}^{\infty }\left[x^{i}\left(k\right)Jx\left(k\right)+r^{i}\left(k\right)cJ\right], \end{array}$$

where the weighting matrix *Q* is

(3) $$\begin{array}{c} Q=\frac{1}{2a^{2}r^{-1}}{\left(\frac{2b^{2}}{a^{2}r^{-1}}p-t\right)}^{-1}\left[a^{2}r^{-1}t^{2}+2\left(1-b^{2}\right)t\right],\\ Q=\frac{1}{2a^{2}r^{-1}}{\left(\frac{2b^{2}}{a^{2}r^{-1}}t-L\right)}^{-1}\left[a^{2}r^{-1}L^{2}+2\left(1-a^{2}\right)L\right]. \end{array}$$

Bring in the parameters and weighting matrix *Q* to get

(4) $$\begin{array}{c} \left(\frac{2b^{2}}{a^{2}r^{-1}}I_{x}-t\right)Q=\frac{1}{2}t^{2}+\frac{1-b^{2}}{a^{2}r^{-1}}t. \end{array}$$

Available through formula

(5) $$\begin{array}{c} Q^{2}+\frac{2\left(1+b^{2}\right)}{a^{2}r^{-1}}Q+\frac{{\left(1+b^{2}\right)}^{2}}{{\left(a^{2}r^{-1}\right)}^{2}}I_{x}={\left(Q+t+\frac{1-b^{2}}{a^{2}r^{-1}}I_{x}\right)}^{2}. \end{array}$$

Virtual reality plays a huge role in military, education, medical treatment, retail, etc., by virtue of its advantages beyond the limitations of time and space and physical conditions, technology is constantly advancing, and virtual reality and reality are constantly merging. The continuous exploration of virtual reality will give mankind more gains and progress. The highest level of virtual reality technology is to achieve human-machine symbiosis. Humans can use self-awareness to directly control machines or complete actions. At this time, virtual reality can be an independent cyberspace, or it can be a reality that is completely integrated with reality. In the context, the equipment can be head-mounted glasses or microimplanted chips. When the human-computer interaction interface changes from a variety of two-dimensional, static, and abstract graphical user interfaces to virtual reality three-dimensional, dynamic, and intuitive natural interfaces, the degree of human-computer interaction is greatly improved, and a new human-computer harmonious relationship will emerge as the times require. And this new human-computer relationship is also an important direction of our scientific and technological development and the continuous prominence of the human subject status to achieve the ultimate goal of virtual reality technology to meet the needs of all aspects of humans [16].

### 2.2. Rehabilitation Treatment of Cerebral Palsy in Children

Cerebral palsy refers to the immature brain of the fetus or infancy caused by various reasons, resulting in movement disorders, postural disorders, and some children with mental retardation. The introduction of rehabilitation in China has not been long, and various technologies are not very mature. Generally speaking, training is aimed at the increase of muscle strength and the decrease of tension in children. Children with cerebral palsy need to recover for a longer time and have a slower ability to solve daily life. Lower limb dysfunction usually leads to uncoordinated movements, poor balance ability, and step abnormal state, increased risk of falling, etc. About 1/3 to 1/2 of hemiplegic patients still have independent walking disorder after 3 months, which is one of the main reasons that affect the ability of daily living of hemiplegic patients. This article consults relevant information and combines the training concept of Lekang classrooms in the city's rehabilitation center, introduces virtual reality technology, trains patients, and combines the two to seek a more effective rehabilitation treatment method for children with cerebral palsy [17].

Abnormal body posture activity and imperfect motor function are the core manifestations of cerebral palsy, and children with cerebral palsy have a certain degree of developmental lag in physical posture and motor function due to different degrees of disease. If you want to understand the degree of cerebral palsy in children with cerebral palsy, it is necessary to formulate a set of objective and scientific evaluation methods and evaluation standards [18].

At present, sports rehabilitation is generally used to rehabilitate children with cerebral palsy. The main aim is to train children with functional tasks so that children with cerebral palsy can adapt to changes in the environment and skills learning in the training process can be used in real life. The main characteristics of the task-oriented training model: first, according to the age of the child, the degree of dysfunction, and the goals that the family members want to achieve, a group of 4–6 people is used as a unit, through group training, collective learning, and motivation of children. Inducing the ability to imitate and compete with each other, so that children can actively challenge difficulties, achieve interaction between individuals and other people, and promote the normal development of personality [19]; second, the focus is to emphasize the initiative of children with cerebral palsy. Exercise, rather than passive or pure auxiliary activities, active learning can achieve greater progress and sense of accomplishment, which is one of the manifestations of normal character development. The task-oriented training mode has the characteristics of intention and rhythm. Intentionalization means that in the training process, it is necessary to master the content of the training that the child can complete. The language of the rehabilitation therapist makes it conscious. By guiding the child to better understand the therapist's intentions, he can complete the action more easily. Rhythm strengthening is mainly to strengthen the sense of rhythm in children, which is of great significance to the improvement of children's motor function, and plays an important role in task-oriented training. Through intentional and rhythmic completion of training, it helps children with cerebral palsy to quickly restore normal motor function [20], shown in Figure 1.

For children to perform task-oriented training, the guidance of the rehabilitation therapist is the key. He must be familiar with the decomposition of an action and be able to tell the children simply and clearly, so that the children can understand and imitate. This training is not a procedure, it is to practice a motor skill as an activity. Rehabilitation therapists need to analyze the movements. One movement may be broken down into several steps, so that the child can perform it step by step and finally combine it [21]. The one-to-many training model of task-oriented training also solves the current problem of more children and fewer rehabilitation therapists and appropriately reduces the pressure on rehabilitation therapists, so that they can face their patients in a better state to achieve twice the result with half the effort effect. The work feature of task-oriented training is to mobilize all resources and abilities that can be mobilized, not for symptoms, but to achieve goals. These goals are determined by social needs. Task-oriented training can allow children to learn comprehensively, not simply to train certain muscle strength and reduce the tension of a certain muscle, but to learn how to complete an action, a task, such as walking and transferring objects. Use a task-oriented training system to promote the personality development of children and master the ability of daily learning and life [22]. In the process of motor learning for children with cerebral palsy, the rehabilitation therapist should explain to the children what they are learning and what their effects are. This can help the children rebuild their brain activities and integrate their movements into their daily lives. The external behavior of children with cerebral palsy can also be improved [23].

### 2.3. Rehabilitation Effect Template

Motor function evaluation plays an important role in the rehabilitation of children with cerebral palsy. On the one hand, the evaluation results can reflect the degree of motor dysfunction in children in real time. On the other hand, it can also assist in clinical diagnosis and guide the formulation of personalized rehabilitation training programs. At present, clinically, motor function scales are mainly used to evaluate children's motor function and rehabilitation training effects, but the current part of the assessment lacks quantitative evaluation standards, and the evaluation results mainly rely on the doctor's experience and subjective feelings [24, 25]. Rehabilitation treatment is the main means to reduce the disability rate, improve the quality of life of patients, and help patients return to their families and society. Recently, some new rehabilitation treatment methods have been gradually applied in clinical applications, such as robot-assisted technology, virtual reality technology, electromyography biofeedback therapy, weight loss walking training, and repetitive transcranial magnetic stimulation, which have achieved good results. In this paper, virtual reality technology is used to parameterize the patient's disease prevention and then transmit it to the data model. The data module receives the needs of users, finds suitable resources through resource evaluation, performs tasks, and completes user requests.

In the current medical environment and actual rehabilitation treatment, how to understand and transform the expectations and needs of users more comprehensively and how to adapt the form, structure and function of products to meet the needs of users is the current focus. Taking into account the resources with the same service function, the attributes of the resources are set according to user preferences and have certain scalability [26], calculated as follows:

(6) $$\begin{array}{c} U_{a}=p*b\frac{j}{i}*c+y-\sum_{m=1}^{m}t. \end{array}$$

In order to calculate the weight of patient attributes and ensure the objectivity of the evaluation results, we use the entropy weight method to determine the entropy value and entropy weight of each resource attribute [27]:

(7) $$\begin{array}{c} t=\frac{1}{\ln\;x}\sum_{n=1}^{1}f_{nm}*\;\ln\;f_{nm},\\ r=\frac{1-\sum_{n=1}^{x}z_{nm}}{y-\sum_{m=1}^{m}t},\\ f_{mn}=\frac{z_{nm\left(r_{nm}-uq_{m}\right)}}{\sum_{n=1}^{x}z_{nm}},\\ \sum_{m=1}^{x}w_{m}=1. \end{array}$$

Set objective weights for each user attribute:

(8) $$\begin{array}{c} d=\sqrt{\sum_{m=1}^{x}w_{n}*{\left(r_{nm}-uq_{m}\right)}^{2}},\\ w_{n}=\frac{1}{1+d\left(r_{n},uq\right)}. \end{array}$$

From this, the matching value *Q* can be obtained:

(9) $$\begin{array}{c} Q_{\delta }=\left\{r_{n}\left|d\;\cos\left(r_{n},uq\right)\right|\geq \delta \right\}. \end{array}$$

Calculate the similarity between the resources in the matching resource set *Q* and the resources requested by the user:

(10) $$\begin{array}{c} \cos\;m\left(r,uq\right)=\alpha *\cos\left(r,uq\right)+\left(1-\alpha \right)*\frac{1}{m}\sum_{n=1}^{m}\delta_{ij}. \end{array}$$

The simulation parameters are calculated as follows:

(11) $$\begin{array}{c} F=\frac{\sum \left(q_{rp,rpn}-q_{rpm}\right)\left(q_{uq,uqn}-q_{uq}\right)}{\sum_{n=1}^{n}{\left(q_{r}-q_{uq}\right)}^{2}\sqrt{\sum {\left(q_{uq,uqm}-q_{uq}\right)}^{2}}}. \end{array}$$

## 3. Virtual Reality Technology in the Rehabilitation of Lower Limb Function of Children with Cerebral Palsy

### 3.1. Experimental Purpose

Through the follow-up investigation of the patients, it was learned whether the pathology of children with cerebral palsy and after treatment, whether the effect of rehabilitation of the lower limb function of children with cerebral palsy was effectively controlled, and whether the control effect was obvious. To study the clinical characteristics and imaging of children with cerebral palsy, summarize and analyze the clinical characteristics, treatment, and prognosis of children with cerebral palsy, and provide reference basis for the early diagnosis, early treatment, and prognosis of children with cerebral palsy.

### 3.2. Experimental Analysis Objects

By collecting the clinical data of children diagnosed with cerebral palsy in the inpatient department of the Children's Hospital of this province (gender, age at diagnosis or diagnosis, clinical symptoms, and signs at admission, auxiliary examinations include seven respiratory virus antigen tests, T lymphocyte subgroup tests, and allergies), routine examinations were performed on these children, including fiberoptic bronchoscopy, BALF cytology counts, lung function tests, and lung CT examinations. In addition, they were followed up through telephone consultation and outpatient clinics. Perform a retrospective analysis of the collected data.

### 3.3. Data Sources

The data in this article are mainly derived from the clinical data of the inpatient diagnosis of the Children's Hospital of the province from 2015 to 2019, as well as the statistics of on-site understanding of patients and telephone interviews. After that, the statistical data are classified and analyzed, and simulated by computer software. We conducted investigations on doctors and patients and asked them to evaluate the effectiveness of the rehabilitation of lower limb function in children with cerebral palsy based on virtual reality technology. The evaluation method was based on the entropy method and comprehensive quantitative and qualitative analysis.

The entropy method is a relatively objective evaluation index weight assignment method, which can effectively avoid the subjectivity of artificial scoring and has high accuracy. However, at the same time, this study also realizes that the entropy method has the defect that it cannot directly reflect the knowledge, opinions, and empirical judgments of experts and scholars, and the weighted results obtained may be contrary to reality. Therefore, this article uses a combination of analytic hierarchy process and entropy method to determine the weight coefficient of each evaluation index of regional higher education.

Quantitative analysis is to analyze the data of the problem, using the intuition and clear essence of mathematics to reflect the existence of the problem; qualitative is to collect, read, organize, and systematically relate the theoretical results of relevant domestic and foreign research documents. Some standards cannot be directly analyzed in a quantitative way but can only be evaluated using a qualitative analysis method. The assessment standard system is constructed using a combination of quantitative and qualitative analysis methods, and formulas related to standard calculations are also given.

## 4. Experimental Analysis of Rehabilitation of Lower Limb Function in Children with Cerebral Palsy

### 4.1. Changes in Children with Cerebral Palsy in Recent Years

We made relevant statistics on all children with cerebral palsy who had been admitted to the hospital from 2010 to 2019 in five hospitals in the province and discussed the trend of changes in children with cerebral palsy in the province. The specific data are shown in Table 1.

From Figure 2, we can see that the number of children with cerebral palsy in our province has shown an upward trend and then a downward trend. It was at the peak of the number of children in 2014 and 2015, but with the continuous improvement of medical technology in recent years, the number of children is declining year by year. We conducted related surveys on hospital doctors and hospital medical records and conducted relevant statistics on the treatment of these children. The specific data are shown in Table 2.

It can be seen from Figure 3 that with the change of time, the number of cured children has increased year by year, and the percentage of cured children has increased from less than 60% in 2010 to about 75%. There may be some factors that the sample size is too small. However, as a whole, the level of medical care and technology is constantly rising, and the level of medical technology and doctors is constantly rising. The cure rate of children with cerebral palsy is increasing year by year.

### 4.2. Age of Children with Cerebral Palsy

We have classified the age of children with cerebral palsy in order to facilitate the classification and formulation of later treatment plans and facilitate rehabilitation treatment. The specific data are shown in Table 3.

From Figure 4, we can see that among the children admitted to the hospital, there are children of all ages, but the age of the main children is between 3 and 10 years old, reaching about 60%, which shows the treatment of children with cerebral palsy. At this time, we must pay attention to the methods and methods of treatment and rehabilitation and fully consider the acceptance level of children of this age to achieve better treatment results.

### 4.3. Changes before and after Treatment in Children with Cerebral Palsy

We treat the children and compare their physical functions before and after treatment, such as upper and lower limb functions, living ability, and balance, make statistics, and use templates to digitize them for easy comparison. The values before treatment are shown in Table 4.

From Figure 5, we can see that the parameters of children with cerebral palsy are very low before treatment, the upper and lower limb function is averaged at about 0.5, and the living ability and balance do not exceed 0.5. At the maximum walking speed of 10 m, it is also far behind a normal child, whose walking speed of 10 meters is about 6 seconds. In order to facilitate comparison, we have made statistics on various parameters of children who have undergone traditional treatment. The specific data are shown in Table 5.

From Figure 6, we can see that after the traditional treatment, the physical function indicators of children with cerebral palsy have improved significantly. For example, in the function of the upper and lower limbs, after the treatment, the functions of the upper and lower limbs of the children are equally divided. It can reach about 0.58, and the balance ability is also about 0.6, which has reached a good level, and the time for the child to walk at the maximum speed of 10 m has also been reduced, reaching about 4.5. For the children based on virtual reality technology, we also conducted 8 weeks of treatment under the virtual technology, and statistics on their various parameters, as shown in Table 6.

From Figure 7, we can see that after 8 weeks of virtual reality technology and treatment, the data of the child have increased a lot compared with the traditional treatment. In terms of upper and lower limb function, the average score can reach more than 0.6. In terms of balance, the score is about 0.7, and in terms of children's exercise, it has basically reached the level of ordinary people, which shows that with the cooperation of virtual reality technology, the lower limb exercise ability of children with cerebral palsy can basically be restored.

## 5. Conclusions

The traditional treatment of children with cerebral palsy mainly relies on one-on-one training by the therapist. The therapist's work intensity is high, and the physical strength requirements of the therapist are high. It is difficult to ensure the continuity and stability of the training; the level of the therapist has a greater impact on the rehabilitation treatment effect. The overall professional quality level of the therapist is relatively high. Rehabilitation training requires one or more rehabilitation therapists to perform rehabilitation training for the patient. However, it is difficult for each therapist to achieve the same method and strength. In the rehabilitation training for the patient, no objective effect evaluation can be obtained; professional venues and equipment are required. Therefore, conventional rehabilitation treatment not only consumes a lot of manpower and time, but the training effect cannot be guaranteed.

There are large differences in the line function status, treatment duration, treatment frequency, duration, training actions, and forms of the existing children with cerebral palsy. Further research is needed to determine the optimal treatment dose, frequency, duration and interventional intervention, and optimal stage, so as to provide patients with the best treatment strategy to achieve the best results. At present, virtual reality technology is mostly used as an auxiliary means of conventional rehabilitation training for research.

At present, there are few studies on children with cerebral palsy in the application of the central nervous system, especially lower limb rehabilitation, but they have improved significantly in the past three years. However, the sample size of many studies is too small and long-term follow-up is lacking. They may affect the experiment persuasiveness of the result. Moreover, virtual reality technology has only appeared in recent years and has not yet reached the stage of technological maturity. These will affect the results of experiments, especially the clinical experience of most relying on therapists, which is difficult to quantify and brings inconvenience to clinical applications. This is also the focus of our future research.

## Figures and Tables

**Figure 1:** Principles of physical education teaching.

**Figure 2:** Changes in the child.

**Figure 3:** Cure of children in recent years.

**Figure 4:** Cure of children in recent years.

**Figure 5:** Cure of children in recent years.

**Figure 6:** Children after treatment.

**Figure 7:** Parameters after virtual reality technology treatment.

**Table 1:** Changes in the number of children.

	2010	2011	2012	2013	2014	2015	2016	2017	2018	2019
First hospital	23	25	19	23	18	19	21	22	21	19
First Affiliated Hospital	20	18	21	19	21	24	22	26	23	17
Provincial University Hospital	19	23	24	25	20	21	20	22	16	18
City People's Hospital	20	23	24	27	24	21	19	17	18	16
Provincial Hospital	21	24	25	26	29	27	23	21	21	18

**Table 2:** Number of children cured.

	2010	2011	2012	2013	2014	2015	2016	2017	2018	2019
First hospital	12	14	13	17	12	16	16	18	19	16
First Affiliated Hospital	13	11	14	16	14	17	14	19	16	12
Provincial University Hospital	11	13	14	17	10	15	16	17	9	13
City People's Hospital	9	12	13	16	11	12	14	11	16	10
Provincial Hospital	11	14	12	14	13	17	15	16	13	15

**Table 3:** Age of child.

	0–2	3–6	7–10	11–12	13–15
First hospital	3	5	2	4	7
First Affiliated Hospital	2	4	3	3	6
Provincial University Hospital	1	6	4	5	7
City People's Hospital	4	9	11	2	5
Provincial Hospital	6	3	5	9	4

**Table 4:** Value before treatment.

	Upper limb ability	Lower limb function	Daily life	Balance	Functional walking classification	10 m maximum walking speed (s)
First hospital	0.43	0.41	0.37	0.47	0.34	5.77
First Affiliated Hospital	0.49	0.46	0.35	0.38	0.48	6.12
Provincial University Hospital	0.44	0.53	0.51	0.47	0.39	6.72
City People's Hospital	0.52	0.58	0.51	0.44	0.47	6.21
Provincial Hospital	0.59	0.62	0.61	0.58	0.49	6.34

**Table 5:** Parameters of children after traditional treatment.

	Upper limb ability	Lower limb function	Daily life	Balance	Functional walking classification	10 m maximum walking speed (s)
First hospital	0.52	0.58	0.51	0.56	0.52	4.47
First Affiliated Hospital	0.59	0.62	0.54	0.61	0.58	4.34
Provincial University Hospital	0.69	0.64	0.68	0.64	0.66	4.21
City People's Hospital	0.75	0.78	0.75	0.76	0.74	4.59
Provincial Hospital	0.79	0.76	0.81	0.73	0.69	4.73

**Table 6:** Virtual reality treatment of children.

	Upper limb ability	Lower limb function	Daily life	Balance	Functional walking classification	10 m maximum walking speed (s)
First hospital	0.58	0.62	0.68	0.69	0.65	3.57
First Affiliated Hospital	0.67	0.61	0.67	0.72	0.62	3.34
Provincial University Hospital	0.65	0.68	0.74	0.78	0.69	3.42
City People's Hospital	0.75	0.77	0.67	0.72	0.74	3.49
Provincial Hospital	0.78	0.82	0.86	0.89	0.87	3.73

## Data Availability

No data were used to support this study.
